This article has been retracted.

# Insulin Aspart Combined with Exercise Therapy in Spleen Deficiency Type Gestational Diabetes Mellitus: The Effect on Disease Control and Pregnancy Outcomes

**DOI:** 10.1155/2022/3084522

**Published:** 2022-05-11

**Authors:** Yingkun Shi, Xueyun Meng

**Affiliations:** Dalian Municipal Women and Children's Medical Center(Group), Dalian City, Liaoning Province 116033, China

## Abstract

**Objective:**

To investigate the effect of insulin aspart combined with exercise therapy on the disease control and pregnancy outcomes of spleen deficiency type gestational diabetes mellitus patients.

**Methods:**

In this prospective study, a total of 102 patients with spleen deficiency type gestational diabetes mellitus admitted to our hospital from January 2019 to December 2019 were selected and assigned at a ratio of 1 : 1 via the random number table method to receive insulin aspart (control group) or insulin aspart plus exercise therapy (observation group). Outcome measures include blood sugar, clinical efficacy, adverse pregnancy outcomes, and complications.

**Results:**

Insulin aspart plus exercise therapy was associated with significantly lower blood glucose and glycosylated hemoglobin levels versus insulin aspart alone (*P* < 0.05). Insulin aspart plus exercise therapy resulted in significantly higher total efficacy (96.08%) versus insulin aspart (74.51%) (*P* < 0.05). Patients receiving insulin aspart plus exercise therapy showed a significantly lower incidence of adverse pregnancy outcomes (3.92%) versus those given insulin aspart alone (37.25%) (*P* < 0.05). Insulin aspart plus exercise therapy resulted in a lower incidence of complications (5.88%) versus insulin aspart (41.17%) (*P* < 0.05).

**Conclusion:**

Exercise therapy plus insulin aspart might offer a viable treatment alternative for patients with spleen deficiency-type gestational diabetes mellitus given its promising effects in disease control and pregnancy outcomes, with good efficacy and safety profiles.

## 1. Introduction

Gestational diabetes mellitus is a common pregnancy complication in the gynecological department. It is an abnormal glucose tolerance disease with a high incidence [1]. For patients with mild diabetes, a reasonable diet and appropriate exercise can control the blood sugar [2, 3]. However, disease progression may be detrimental to the mother and the fetus, resulting in adverse consequences such as gestational hypertension, miscarriage, and neonatal asphyxia [4, 5]. Traditional Chinese medicine believes that the onset of gestational diabetes is associated with spleen deficiency and poor diet, and treatment aims to strengthen the spleen, promote fluid production, benefit qi, and nourish yin [4]. Accordingly, effective measures for the management of blood glucose levels without compromising health are essential to ensure the safety of the mother and fetus. The causes of spleen deficiency type gestational diabetes include age, obesity, stress, and genetic factors. Currently, insulin resistance and pancreatic *β*-cell secretion dysfunction are considered the main contributors to gestational diabetes, which is treated clinically with diet-exercise therapy and insulin intervention. Diet-exercise therapy is the development of a reasonable diet and exercise program for patients to control blood glucose by means of controlled diet and exercise [6–9]. Menthol insulin is a drug commonly used clinically to treat gestational diabetes and has been reported to significantly reduce blood glucose and glycosylated hemoglobin concentrations in patients with gestational diabetes [10, 11]. It has been found that insulin combined with individualized diet for the treatment of gestational diabetes can achieve better outcomes compared with single treatment [12]. Nevertheless, the synergy of insulin aspart and exercise in gestational diabetes mellitus has been marginally explored. This study was designed to investigate the effect of insulin aspart plus exercise therapy on patients with gestational diabetes mellitus.

## 2. Study Design and Participants

### 2.1. Participants Profile

In this prospective study, a total of 102 patients with gestational diabetes mellitus admitted to our hospital within one year (2019) were enrolled and assigned (1 : 1) via the random number table method to either a control group or an observation group. The patients in the control group were 24–32 years old, and those in the observation group were 23–33 years old. All were singleton pregnancy. The two groups showed similar baseline data. The study was approved by the Ethics Committee of the Dalian Municipal Women and Children's Medical Center (Group) and all patients gave their informed consent.

### 2.2. Inclusion and Exclusion Criteria

#### 2.2.1. Inclusion Criteria

The inclusion criteria were as follows: patients with a diagnosis conforming to the diagnostic guidelines and standards for gestational diabetes [6], with no allergies or contraindications to the drugs in the study, lung, stomach, spleen, kidney, and the pathogenesis was yin deficiency, and weak qi is the essence, and heat and blood stasis are the symptoms.

#### 2.2.2. Exclusion Criteria

The exclusion criteria were as follows: with complications during pregnancy, with vital tissues and organs dysfunction such as the heart and lungs, and with the withdrawal of consent.

The participants all provided written informed consent after being fully informed of the process and the purpose of the study.

### 2.3. Treatment Methods

Both groups were given the methods of clearing the lungs and venting the stomach, purging the fire and preserving the body fluid; nourishing the lungs and invigorating the kidneys, nourishing the water and promoting the body fluid; strengthening the spleen to help transport, invigorating qi, and transforming Jinmen; removing blood stasis and dredging collaterals and blood circulation. Shenqi Maiwei Dihuang decoction, 20 g of *Astragalus*, 15 g each of Taizishen, *Ophiopogon japonicus*, 12 g each of Chinese yam, *Schisandra*, *Poria*, and 10 g each of *Rehmannia glutinosa*, *Cornus*, *Alisma*, Cortex Moutan, and licorice, 1 dose per day, boiled with water, 150 ml of soup each time, administered in the morning and in the evening for 4 weeks.

The patients in the control group received insulin aspart (State Drug Certificate J20150073), and the patients in the observation group were treated with insulin aspart (State Drug Certificate J20150073) plus exercise therapy, and the specifics are as follows: the initial dose of insulin aspart was controlled at 0.2 IU/(kg·d) and then was adjusted depending on patients' blood sugar changes [8]. The patients were instructed to carry out moderate aerobic exercise in daily life to ensure sufficient daily activity. Exercise is mainly simple and low to medium intensity aerobic exercise, such as running in place, walking, alternate lifting, and stair climbing, performed after meals. The intensity of exercise could be gradually increased from 10 min/time to 30 min/time, with a break of about 5 min in between, 3-4 times/week. The exercises were promptly discontinued in the event of discomfort, and medical attention was sought if necessary [9, 10].

### 2.4. Outcome Measures

Blood sugar: 2–4 ml of fasting venous blood was collected before treatment, after treatment, and two hours after meals, and the blood sugar levels of the two groups of patients were analyzed and compared, including fasting blood sugar (FPG), 2 h postprandial blood sugar (2hPBG), and glycated hemoglobin (GHb). 2 tubes of fasting venous blood of 2 mL each were collected from all study subjects, one tube was centrifuged for the determination of fasting blood glucose, and the other was anticoagulated with EDTA-K2 to determine glycated hemoglobin. Patients ate 100 g steamed bread meal, and 2 mL of venous blood was collected 2 h later for measurement of 2 h postprandial glucose, and the determination method was the same as that of fasting glucose. The blood glucose testing instrument was the Olympus AU640 automatic biochemical analyzer, and the reagents were provided by Shanghai Rongsheng Biological Pharmaceutical Co. Blood glucose was determined by the glucose oxidase method. Glycosylated hemoglobin was determined by high performance liquid chromatography (HPLC) using a Bio-Rad 10 glycosylated hemoglobin analyzer from the United States, and standards and quality control products were provided by Landau, UK.

Clinical efficacy: Markedly effective: the symptoms and signs were significantly alleviated, and test indicators after treatment returned to a normal level. Effective: the symptoms and signs were alleviated, and the test indicators after treatment showed significant improvement. Ineffective: no improvement or aggravation occurs after treatment.

Adverse pregnancy outcomes: Adverse pregnancy outcomes such as premature rupture of membranes, postpartum hemorrhage, and postpartum infection were counted and compared.

Complications: the incidence of neonatal complications was calculated and analyzed, including macrosomia, respiratory distress syndrome, and neonatal hypoglycemia.

### 2.5. Statistical Analysis

All data analyses were performed with the software SPSS 22.0. The measurement data were expressed as (x ± s) and processed via the independent sample *t*-test. The enumeration data were expressed as the rate (%) and examined via the chi-square test. Differences were considered statistically significant at *P* < 0.05.

## 3. Results

### 3.1. Baseline Features

The baseline features of the control group (aged 24–39 years, gestational age of 15–30 weeks) were comparable with those of the observation group (aged 25–41 years, gestational age of 15–19 weeks) (*P* > 0.05) (Table 1).

### 3.2. Blood Glucose and Glycosylated Hemoglobin Levels

Before treatment, there was no significant difference in FPG, 2hPBG, and GHb between the observation group and the control group (*P* > 0.05). Insulin aspart plus exercise therapy was associated with significantly lower levels of FPG, 2hPBG, and GHb versus insulin aspart alone (*P* < 0.05, Table 2).

### 3.3. Clinical Efficacy

Insulin aspart plus exercise therapy resulted in significantly higher total efficacy (96.08%) versus insulin aspart (74.51%) (*P* < 0.05, Table 3).

### 3.4. Pregnancy Outcomes

#### 3.4.1. Adverse Pregnancy Outcomes of Patients

Patients receiving insulin aspart plus exercise therapy showed a significantly lower incidence of adverse pregnancy outcomes (3.92%, including 1 case of excessive amniotic fluid and 1 case of postpartum hemorrhage) versus those given insulin aspart alone (37.25%, including 4 cases of excessive amniotic fluid, 3 cases of premature fetal membrane compression, 8 cases of postpartum hemorrhage, and 4 cases of postpartum infection) (*X*^2^ = 17.33, *P* < 0.05).

### 3.5. Neonatal Complications

Insulin aspart plus exercise therapy resulted in a lower incidence of complications (5.88%, including 1 case of gigantism, 1 case of hypoglycemia, and 1 case of prematurity) versus insulin aspart (41.17%, including 4 cases of gigantism, 7 cases of hypoglycemia, 7 cases of prematurity, and 3 cases of respiratory distress syndrome occurred) (*X*^2^ = 17.654, *P* < 0.05).

## 4. Discussion

Gestational diabetes mellitus is defined as diabetes developed during pregnancy, with the normal glucose metabolism or potential impaired glucose tolerance before pregnancy. The global incidence is 1–14% and in China is about 1–5% and has been on a rise in recent years [11]. The main presentations include dry mouth, polydipsia, polyphagia, and body weight loss, and symptoms of the itchy skin can also be seen in some cases. It compromises the growth and development of the fetus, which necessitates early intervention to control blood sugar [12]. At present, exercise therapy and insulin are widely used in clinical intervention for gestational diabetes mellitus [13, 14]. Studies have found that insulin aspart can significantly reduce blood glucose and glycosylated hemoglobin concentrations in patients with gestational diabetes mellitus [15, 16]. To the best of our knowledge, exercise therapy is exercise program tailored based on the patient's conditions to help them control their blood sugar [17, 18]. Previous research has demonstrated that insulin combined with individualized exercise gains promising results in the treatment of gestational diabetes [19].

MicroRNAs (miRNAs) are factors that regulate biological functions and participate in biological processes such as cell division, proliferation, differentiation, and development. Recent studies have shown that miRNAs are also involved in the regulation of adipocyte differentiation, glucose and lipid metabolism, energy homeostasis, and insulin production and secretion, suggesting that such small nucleic acid molecules may be involved in the pathogenesis of metabolic diseases such as obesity and diabetes [20]. The expression of miRNA-143 in the placenta tissue of patients with gestational diabetes increased, suggesting that miRNA-143 may be related to the pathogenesis of patients with gestational diabetes and that exercise can reduce the expression of miRNA-143 in patients with gestational diabetes and help reduce blood sugar in patients with gestational diabetes [21]. The results of the present study showed that insulin aspart plus exercise therapy was associated with significantly lower levels of FPG, 2hPBG, and GHb versus insulin aspart alone. Insulin aspart is a fast-acting insulin, with a similar drug activity to that of natural insulin that can maintain the blood sugar level in a reasonable and stable range in the long run. Additionally, the combination of exercise therapy promotes the digestive function of patients and increases the metabolism of carbohydrates to achieve blood sugar control of patients.

Moreover, the present study reported a higher clinical efficacy of insulin aspart plus exercise therapy versus monotherapy of insulin aspart. The insulin was administered via subcutaneous injection, which ensures the effectiveness of the drug as well as potency duration. Notably, in terms of pregnancy outcome and neonatal complications, the combined therapy also outperformed the monotherapy because the reason can be that insulin aspart plus exercise therapy improves the patient's systemic blood circulation, reduces insulin resistance, controls the body's blood sugar, and minimizes the impact on pregnant women and fetuses, thus reducing the incidence of complications during pregnancy [20]. It further indicates that the combination therapy benefits the control of gestational diabetes mellitus and contributes to a lower incidence of pediatric complications.

Shenqi Maiwei Dihuang decoction is composed of *Astragalus*, *Radix pseudostellariae*, Ophiopogonis Radix, prepared *Rehmannia* root, Chinese yam, *Cornus officinalis*, *Schisandra*, Alismatis Rhizoma, *Poria*, Moutan Cortex, and licorice, which are effective in strengthening the spleen, benefiting qi, nourishing yin, and moistening dryness. This formula clears heat, nourishes yin, benefits qi, generates fluid, strengthens the spleen, and tonifies the kidney, which is consistent with the treatment of qi and yin deficiency in gestational diabetes mellitus in Chinese medicine. Modern pharmacological research has found that *Astragalus* can enhance immunity, improve the material metabolism, regulate blood glucose levels, and inhibit oxygen-free radicals. *Radix pseudostellariae* can regulate immunity, promote antioxidation, lower blood sugar, and promote microcirculation. Ophiopogonis Radix can enhance immunity, improve the body's adaptability, and has a certain hypoglycemic effect. Prepared *Rehmannia* root Radix Rehmanniae is anti-inflammatory, diuretic, and hypoglycemic. The Chinese yam is anti-inflammatory and hypoglycemic and prevents lipid deposits in blood vessel walls. *Cornus officinalis* can enhance immunity and reduce inflammation, with antibacterial and antioxidant effects. *Schisandra* can reduce inflammation, enhance immunity, and eliminate free radicals. Alismatis Rhizoma is diuretic and hypolipidemic. *Poria* can enhance immunity with antibacterial and antitumor effects and also protect the liver. Moutan Cortex has antiatherosclerosis, diuretic, and anti-inflammatory effects. Licorice can enhance immunity with antibacterial and anti-inflammatory properties.

## 5. Conclusion

Exercise therapy plus insulin aspart might offer a viable treatment alternative for patients with gestational diabetes mellitus given its promising effects in disease control and pregnancy outcomes, with good efficacy and safety profiles.

## Figures and Tables

**Table 1:** Comparison of general data between two groups of patients.

Group	Age	Gestational age	Primipara	Multiparous
Observation group	28.69 ± 4.12	23.9 ± 4.4	40	11
Control group	27.71 ± 3.65	23.4 ± 4.7	38	13
*t*/*X*^2^	1.365	2.647	4.265	
*P*	0.415	0.741	0.241	

**Table 2:** Comparison of blood glucose and glycated hemoglobin levels before and after treatment in the two groups ($\bar{\text{x}}$ ± s).

Groups	*n*	Before treatment			After treatment		
		FPG (mmol/L)	2hPBG (mmol/L)	GHb (%)	FPG (mmol/L)	2hPBG (mmol/L)	GHb (%)
Observation group	51	6.82 ± 1.01	8.18 ± 2.07	6.23 ± 1.33	5.01 ± 0.39	6.85 ± 0.44	5.01 ± 0.23
Control group	51	6.68 ± 1.27	8.21 ± 1.89	6.30 ± 1.29	5.99 ± 0.95	7.02 ± 0.42	6.23 ± 0.58
*t*	—	0.616	0.076	0.270	6.815	1.996	13.964
*P*	—	0.539	0.940	0.788	＜0.001	0.049	＜0.001

**Table 3:** Comparison of clinical efficacy between the two groups of patients (*n* (%)).

Groups	*n*	Markedly effective	Effective	Ineffective	Total
Observation group	51	21	28	2	96.08
Control group	51	14	22	13	74.51
*X* ^2^	—	—	—	—	9.457
*P*	—	—	—	—	0.002

## Data Availability

The data generated or analyzed during this study are included within the article.
